The article "Serum Epitope Repertoire Analysis Enables Early Detection of Lyme Disease with Improved Sensitivity in an Expandable Multiplex Format" was published in 2021. Journal: J Clin Microbiol.

# Serum Epitope Repertoire Analysis Enables Early Detection of Lyme Disease with Improved Sensitivity in an Expandable Multiplex Format

**DOI:** 10.1128/JCM.01836-20

**Published:** 2021-01-21

**Authors:** Jack Reifert, Kathy Kamath, Joel Bozekowski, Ewa Lis, Elizabeth J. Horn, Dane Granger, Elitza S. Theel, John Shon, Jaymie R. Sawyer, Patrick S. Daugherty

**Affiliations:** a Serimmune Inc., Goleta, California, USA; b Lyme Disease Biobank, Portland, Oregon, USA; c Division of Clinical Microbiology, Department of Laboratory Medicine and Pathology, Mayo Clinic, Rochester Minnesota, USA; University of Tennessee at Knoxville

**Keywords:** Lyme disease, antibody repertoire, immunoserology, serology

## Abstract

Widely employed diagnostic antibody serology for Lyme disease, known as standard two-tier testing (STTT), exhibits insufficient sensitivity in early Lyme disease, yielding many thousands of false-negative test results each year. Given this problem, we applied serum antibody repertoire analysis (SERA), or next-generation sequencing (NGS)-based serology, to discover IgG and IgM antibody epitope motifs capable of detecting Lyme disease-specific antibodies with high sensitivity and specificity. Iterative motif discovery and bioinformatic analysis of epitope repertoires from subjects with Lyme disease (*n* = 264) and controls (*n* = 391) yielded a set of 28 epitope motifs representing 20 distinct IgG antibody epitopes and a set of 38 epitope motifs representing 21 distinct IgM epitopes, which performed equivalently in a large validation cohort of STTT-positive samples. In a second validation set from subjects with clinically defined early Lyme disease (*n* = 119) and controls (*n* = 257), the SERA Lyme IgG and IgM assay exhibited significantly improved sensitivity relative to STTT (77% versus 62%; Z-test; *P* = 0.013) and improved specificity (99% versus 97%). Early Lyme disease subjects exhibited significantly fewer reactive epitopes (Mann-Whitney U test; *P* < 0.0001) relative to subjects with Lyme arthritis. Thus, SERA Lyme IgG and M panels provided increased accuracy in early Lyme disease in a readily expandable multiplex assay format.

## Abstract (precis)

Widely employed diagnostic antibody serology for Lyme disease, known as standard two-tier testing (STTT), exhibits insufficient sensitivity in early Lyme disease, yielding many thousands of false-negative test results each year. Given this problem, we applied serum antibody repertoire analysis (SERA), or next-generation sequencing (NGS)-based serology, to discover IgG and IgM antibody epitope motifs capable of detecting Lyme disease-specific antibodies with high sensitivity and specificity. Iterative motif discovery and bioinformatic analysis of epitope repertoires from subjects with Lyme disease (*n* = 264) and controls (*n* = 391) yielded a set of 28 epitope motifs representing 20 distinct IgG antibody epitopes and a set of 38 epitope motifs representing 21 distinct IgM epitopes, which performed equivalently in a large validation cohort of STTT-positive samples.

The article "Serum Epitope Repertoire Analysis Enables Early Detection of Lyme Disease with Improved Sensitivity in an Expandable Multiplex Format" was published in 2021. Journal: J Clin Microbiol.

## INTRODUCTION

Lyme disease caused by Borrelia burgdorferi remains the most common vector-borne disease in the United States (1), with rising incidence and prevalence (2). Prompt diagnosis and treatment during early stages of infection typically result in resolution without apparent prolonged symptoms and positive outcomes (3, 4). However, a substantial fraction of those infected do not receive timely diagnosis or effective therapy and experience symptoms, including cardiac-related complications, musculoskeletal symptoms, pain and peripheral neuropathy, and memory loss (4). The economic costs of untreated and late Lyme disease in the United States have been estimated at $25 to $75 billion (5). Even so, since B. burgdorferi is just one of many tick-borne pathogens (6), these numbers may underestimate the full impact of tick-borne disease-associated health care costs.

The diagnosis of Lyme disease is aided by detection of antibodies to B. burgdorferi using the standard two-tier testing (STTT) algorithm, which incorporates a first-tier enzyme immunoassay (EIA) and second-tier IgG and/or IgM immunoblotting (7) or a variation of this algorithm known as modified two-tier testing (MTTT), replacing the second-tier immunoblot with a second enzyme-linked immunosorbent assay (ELISA) (8). False-negative results frequently arise from insufficient antibody concentrations during early localized disease, causing reduced sensitivity (9, 10). Meanwhile, IgM immunoblots used in STTT to detect early Lyme disease exhibit nonoptimal specificity, leading to frequent false-positive tests (11), unnecessary antibiotic use, and delayed diagnosis of other conditions with symptoms similar to Lyme disease. These problems prompted national efforts to assemble specimen biobanks and develop new diagnostic tools to improve early disease detection (8, 12). As a result, several novel assays have been developed and exhibit improved performance (13, 14). Meanwhile, recognition of the high burden of non-Lyme tick-borne infections, either alone or in combinations, including babesiosis, anaplasmosis, and rickettsioses (6), has spurred development of multiplex tests, for example, using solid-phase peptide arrays (15). Despite these efforts, there remains a significant unmet need for accurate multiplex tests that reveal the full burden of tick-borne infections across all stages of disease.

The article "Serum Epitope Repertoire Analysis Enables Early Detection of Lyme Disease with Improved Sensitivity in an Expandable Multiplex Format" was published in 2021. Journal: J Clin Microbiol.

We previously described a next-generation sequencing (NGS)-based serology platform enabling discovery of antigenic epitopes, with effectively unlimited multiplexing, termed serum epitope repertoire analysis (SERA) (16). SERA integrates high-diversity random peptide libraries (16), NGS, and bioinformatic tools and computational analytics (17–19) to discover a multitude of pathogen-specific antibody epitopes and optimize their combinations to create high-performance serology tests (16). Application of SERA to specimens from subjects with chronic Chagas disease resulted in an IgG assay exhibiting 100% sensitivity with 99.6% specificity (16), exceeding the performance of current parallel independent tests required to achieve high specificity (20). Because SERA uses a library of ∼10 billion random peptides that can effectively mimic nearly any protein-based antigen, the high-content archival data sets that SERA generates can be analyzed for antibodies associated with many different infections (21), allergies, and autoimmune diseases (19, 21). Given the potential to create an accurate multiplex test for tick-borne diseases and other diseases with overlapping symptoms, we applied SERA to develop an assay for Lyme disease with improved diagnostic accuracy. Our results elucidate both characterized and novel antigenic epitopes giving improved sensitivity and specificity relative to STTT, and provide a path to an accurate, comprehensive, and expandable tick-borne disease assay.

## MATERIALS AND METHODS

### Biospecimens.

Deidentified specimens along with associated Lyme disease testing data used in this study are listed (Table 1). Specimens provided from the CDC biorepository and Mayo Clinic include the following cohorts: discovery Lyme (*n* = 222), validation Lyme (*n* = 454), and confirmed negative discovery controls (*n* = 39). Table 1 lists all clinically defined Lyme disease and control samples provided by the CDC and LDB used to compare SERA to the standard two-tier testing (STTT) algorithm. The inclusion criteria and testing for the provided clinical samples were previously defined in detail from the CDC (9) and the LDB (12). Untested, presumed non-Lyme validation controls (*n* = 1,076) representing multiple other infections and disorders as well as healthy donors were sourced from commercial vendors.

**TABLE 1:** Biospecimen cohorts used in this study^*a*^

Cohort	Source	No. of specimens	STTT result (%)			
			Negative	IgG+^*b*^	IgG+, IgM+^*b*^	IgM+^*b*^
Lyme disease discovery cohort	MC	222	0 (0)	96 (43)	13 (6)	113 (51)
Lyme disease validation cohort	MC	454	0 (0)	97 (21)	163 (36)	194 (43)
Controls						
Discovery cohort (tested)^*d*^	CDC	39	36 (92)	0 (0)	0 (0)	3 (8)
Discovery cohort (untested)	Commercial	391	NA	NA	NA	NA
Validation cohort (untested)	Commercial	1,076	NA	NA	NA	NA
Clinically defined Lyme^*c*^	CDC	71				
Lyme arthritis, carditis, neuroborelliosis		37	0 (0)	20 (54)	13 (35)	4 (11)
Acute		34	20 (59)	3 (9)	4 (12)	7 (21)
Convalescent (matched)		34	10 (29)	5 (15)	7 (21)	12 (35)
Clinically defined Lyme	LDB	48				
Early		25	13 (52)	1 (4)	4 (17)	7 (30)
Acute		23	13 (52)	2 (9)	0 (0)	9 (39)
Convalescent (matched)		23	10 (43)	1 (4)	4 (17)	8 (35)
Clinically defined controls	CDC	131				
Endemic, nonendemic^*d*^		53	53 (100)	0 (0)	0 (0)	0 (0)
Mononucleosis^*d*^		21	18 (86)	0 (0)	0 (0)	3 (14)
Fibromyalgia		16	16 (100)	0 (0)	0 (0)	0 (0)
Multiple sclerosis		11	11 (100)	0 (0)	0 (0)	0 (0)
Rheumatoid arthritis		10	10 (100)	0 (0)	0 (0)	0 (0)
Syphilis		10	9 (90)	0 (0)	0 (0)	1 (10)
Periodontitis		10	9 (90)	0 (0)	0 (0)	1 (10)
Clinically defined controls	LDB	126	124 (98)	1 (1)	0 (0)	1 (1)

a Abbreviations: CDC, Centers for Disease Control and Prevention; LDB, Lyme Disease Biobank; MC, Mayo Clinic; NA, not applicable.

b IgG+, IgG positive; IgM+, IgM positive.

c Forty-two clinically defined Lyme disease samples were included into Lyme panel discovery.

d Nineteen endemic and nonendemic samples plus twenty mononucleosis control samples were included in the Lyme panel discovery.

The article "Serum Epitope Repertoire Analysis Enables Early Detection of Lyme Disease with Improved Sensitivity in an Expandable Multiplex Format" was published in 2021. Journal: J Clin Microbiol.

### IgG and IgM epitope repertoire screening.

Serum specimens were screened for IgG specificities against a fully random Escherichia coli expressed 12-mer peptide library with an estimated diversity of 10^10^ as described previously (16). For IgM isotype screening, the protocol was adjusted as follows: (i) after serum incubation with the library, E. coli cells were centrifuged, the supernatant was removed, and the cells were resuspended in 500 μl 1× phosphate-buffered saline (PBS) containing a 1:100 dilution of biotin-SP (long spacer)-conjugated donkey anti-human IgM secondary antibody (Jackson ImmunoResearch; catalog no. 709-066-073); (ii) the plate was incubated for 1 h at 4°C with orbital shaking (800 rpm), the cells were again centrifuged, supernatant was removed, and cells were resuspended in 900 μl of 1× PBS plus 100 μl of Dynabeads MyOne streptavidin T1-coated magnetic beads (Thermo Fisher Scientific; catalog no. 65601); and (iii) the plate was incubated for 1 h at 4°C with orbital shaking (800 rpm), after which time the plate was magnetized and the bead-antibody complex, along with their bound peptide-bearing cells, were captured. Unbound cells in the supernatant were removed, and the beads were resuspended in 1 ml of 1× PBS to serve as a wash. In this manner, the beads were washed 5 times before growth medium was added and the retained E. coli cells were grown overnight. All subsequent steps were identical for IgG and IgM screening as described previously (16).

The article "Serum Epitope Repertoire Analysis Enables Early Detection of Lyme Disease with Improved Sensitivity in an Expandable Multiplex Format" was published in 2021. Journal: J Clin Microbiol.

### NGS and antibody epitope repertoire generation.

Following amplicon NGS of selected IgG or IgM library members, a nonredundant peptide list of antibody binding epitopes was generated using publicly available software as described previously (21). FASTQ DNA sequencing files were deposited into the NCBI Sequence Read Archive (SRA) for public access. Sequence processing was performed as described previously to yield a unique list of IgG and IgM binding peptides (antibody epitope repertoire) for each specimen (21).

### Lyme disease diagnostic IgG and IgM motif panel creation.

Lyme disease-specific motifs were discovered from the IgG and IgM epitope repertoires using the IMUNE computational algorithm (21). A subset of 20 to 30 samples from the discovery Lyme cohort (*n* = 222) was iteratively used for discovery to identify patterns enriched in at least 25% of the Lyme samples used but not in discovery controls (*n* = 39) (100% specificity). To aid in epitope discovery, particularly toward early Lyme samples, a subset of the CDC clinical cohort samples was included in the iterative IMUNE analysis. These samples are listed as follows: disease group, which includes Lyme arthritis (*n* = 22, stage 3) and acute early Lyme (*n* = 20, stage 1) samples, of which 7 were STTT negative; and the control group, which includes endemic (*n* = 9), nonendemic (*n* = 10), and mononucleosis controls (*n* = 20). Here, a pattern refers to 5 to 10 amino acids wherein five amino acids are defined and the remaining positions are denoted as *x* for any amino acid. Patterns were aligned to generate motifs which can include multiple amino acids at any given position denoted by brackets. Motif enrichment values were standardized using

$$z_{i}=\frac{x-\text{μ}}{\text{σ}}$$

where *z_i_* is the z-score of motif *i*, *x* is the motif enrichment within a repertoire, μ is the average enrichment of control cohort, and σ is the standard deviation for motif *i* in the control cohort. A Z-score of ≥ 4 was considered positive for motif-specific sensitivity and specificity calculations. Motifs were down-selected if they were not positive for any samples or positive in only a few disease samples not used for IMUNE and/or when motifs showed a specificity of < 98% in an untested discovery control cohort (*n* = 391).

Motifs that represented the same or an overlapping epitope were grouped, and where possible, the motif with the greatest sensitivity and mean enrichment was selected for inclusion into the Lyme panel. In several cases, two or more motifs were selected from the same group in order to improve panel sensitivity (Table S1 in the supplemental material). A “composite score” of arbitrary units (AU) was calculated as the sum of the normalized scores (*z_i_*) for each panel (using the maximum motif z-score for groups). A composite score value for the IgG motif panel ≥28 or for the IgM motif panel ≥35 was used as the diagnostic criteria for Lyme disease.

The article "Serum Epitope Repertoire Analysis Enables Early Detection of Lyme Disease with Improved Sensitivity in an Expandable Multiplex Format" was published in 2021. Journal: J Clin Microbiol.

### Identification of candidate antigens.

Panel motifs were queried against the B. burgdorferi proteome using ScanProsite (UniProt/TrEMBL) to generate a list of candidate antigens (multiple strains queried). Example IgG and IgM candidate antigens are provided along with motif-specific sensitivity and specificity values calculated using the validation Lyme and validation control cohorts.

### Statistics.

SERA performance was compared to STTT in the combined LDB and CDC clinical Lyme cohorts. Sensitivity, specificity, and overall accuracy were compared using a proportions test (Z-test) for the total number of correctly called samples within the population size. *P* values are provided for each comparison in the Results section, and 95% confidence interval ranges are provided as error bars or listed where appropriate. When comparing the number of positive motifs between Lyme arthritis samples and the acute- and convalescent-phase samples, a Mann-Whitney test was used.

### Data availability.

All relevant data are included within the manuscript and supplementary tables and the unique peptide sequence sets revealed by bacterial display peptide library selection and NGS for each specimen are available upon request to the authors.

## RESULTS

To identify conserved immunogenic epitopes of IgG and IgM antibodies specific for Lyme disease, we analyzed 222 serum samples from individuals who are STTT positive for Lyme disease (Lyme disease discovery cohort), as well as 42 serum samples clinically defined by the CDC as having Lyme disease using multiple sets of criteria, including erythema migrans (EM), molecular biology testing, and STTT (9). The CDC cohort used in motif discovery included 22 STTT-positive Lyme arthritis samples (stage 3) and 20 matched acute and convalescent early Lyme samples (stage 1), of which 4 were STTT negative. Also included in discovery were sera from individuals without Lyme disease (*n* = 39), which included 9 endemic and 10 nonendemic controls and 20 specimens from individuals with mononucleosis (9) (Table 1). Specimens were processed using the SERA assay workflow (16) in a 96-well plate format by (i) incubation of serum with the peptide library and separation of IgG or IgM antibody-binding library members using conjugated magnetic beads; (ii) growth of the selected library, plasmid isolation, and barcoded PCR amplification of the peptide-encoding regions for each specimen; and (iii) pooling and sequencing of the amplicon libraries using NGS. The unique set of antibody-binding peptides for each specimen, or “epitope repertoires,” were compiled for computational analysis (Fig. 1).

The article "Serum Epitope Repertoire Analysis Enables Early Detection of Lyme Disease with Improved Sensitivity in an Expandable Multiplex Format" was published in 2021. Journal: J Clin Microbiol.

**FIG 1:** The SERA assay workflow. In step 1, serum antibodies interact with antigen mimics displayed on the surface of bacteria allowing for capture of those bacteria. In step 2, the plasmid encoding the peptides that serve as the antigen mimics are amplified from the plasmids, and sample-specific sets are barcoded for NGS. In step 3, motif epitopes are identified that represent antigens for disease-specific antibodies.

Epitope motif discovery was performed using IMUNE, a custom bioinformatic algorithm that has been described in detail elsewhere (21). IMUNE analysis of the repertoires from Lyme disease specimens and controls produced between 100 and 300 candidate motifs for both IgG and IgM assays, depending on the specific samples used. Iterative IMUNE discovery generated a total of >500 candidate motifs, which were ranked based on specificity among 391 additional epitope repertoires (discovery controls) derived from individuals not tested for Lyme disease (Table 1). Motifs that were significantly enriched in more than 7/391 controls were removed to obtain panels of highly specific motifs corresponding to conserved antigenic epitopes of B. burgdorferi proteins that varied among individuals and across disease stages (Fig. 2). The resulting IgG and IgM panels were comprised of 28 motifs representing 20 distinct epitopes and 38 motifs representing 21 epitopes, respectively (Tables S1 and S2 in the supplemental material, respectively).

**FIG 2:** Lyme disease panel motif enrichments. Enrichment of Lyme disease-specific motifs within the peptide epitope repertoires obtained from Lyme disease samples (*n* = 140) and control (*n* = 260) from the discovery set. Lyme groups indicated include LA, Lyme arthritis; acute, early Lyme draw; and IgM, IgM STTT positive.

Lyme disease-specific motifs were mapped to candidate antigens in the Swiss-Prot/TrEMBL database using the ScanProsite search engine (22) (Table 2). Many motifs mapped to known antigens, including variable large protein (VlsE), flagellar, and p66 proteins. For the IgG panel, 11 of 28 motifs mapped to multiple sites within the VlsE antigen and were highly sensitive and specific for Lyme disease (Table 2). Additionally, some motifs mapped to antigens that are less well characterized (Table 2). For example, the motif [IVL]x[LI]xxM[DSE]K mapped to lipoprotein MlpB, an outer membrane protein that may contribute to pathogenesis (23). While hundreds of motifs were identified within ∼150 candidate B. burgdorferi antigens, a small subset of these motifs met our stringent specificity criteria (>98%). Notably, some motifs mapped to known antigens such as OspB, OspC, and p22 but were not included in the final panel due to reduced specificity among discovery controls and a lack of improved sensitivity among our Lyme disease discovery cohort.

The article "Serum Epitope Repertoire Analysis Enables Early Detection of Lyme Disease with Improved Sensitivity in an Expandable Multiplex Format" was published in 2021. Journal: J Clin Microbiol.

**TABLE 2:** Selected Borrelia burgdorferi-specific motifs with candidate antigens and epitopes

Isotype	Motif	Candidate antigen	Candidate epitope	Sensitivity (%)	Specificity (%)
IgG	[KR]x[DE]xTNxF	Variable large protein (VlsE)	KDDPTNkF	26	99.0
	[DA]DPTN	Variable large protein (VlsE)	KDDPTNkF	27	99.2
	[LI]xxA[ILV]xxRG	Variable large protein (VlsE) (2 repeats)	IaaAIalRG	63	99.6
	[DN][AS]A[AG]F	Variable large protein (VlsE)	NAAAF	20	99.8
	VQQExxxxxP	Flagellar filament 41-kDa core protein (flagellin)	QEGVQQEgaqqqP	19	99.9
	QEG[IV]Q	Flagellar filament 41-kDa core protein (flagellin)	QEGVQQEgaqqqP	31	99.4
	Q[TI]EQxxxxxK	Integral outer membrane protein P66	QTEQsststK	16	99.9
	PFx[AP]YxK	Integral outer membrane protein P66	PFsAYiK	14	97.8
	IPxxV[IF]xxR	PF32 plasmid partition protein	IPifVIitR	34	99.7
IgM	[KM]xxxSM[DE]K	Virulent strain-associated repetitive antigen A (VraA protein)	KyvkSMEK	10	98.6
	KTCC	Putative antigen P35	plKTCCdhi	12	99.7
	QQE[GA][AV]	Flagellar filament 41 kDa core protein (flagellin)	QQEGA	15	99.7
	[IVL]x[LI]xxM[DSE]K	Lipoprotein MlpB	IiItnMEK	21	99.2
	[LIP][QN][VRKI]PF	GlpE protein	INIPF	6	99.2

To utilize the full set of motifs for disease classification, a composite score was calculated by summing the standardized enrichment values for each motif as described (16) (see Materials and Methods). A cutoff for positivity was set to achieve an overall specificity of 99.5% among the discovery controls. Together, the Lyme IgG and IgM motif panels exhibited an 87.8% (95% confidence interval [CI], 83.5 to 92.1%; 195/222) positive agreement to STTT in the Lyme disease discovery cohort (Fig. 3).

**FIG 3:** Sample scores on Lyme IgG and IgM motif panels. (A) Discovery and validation specimen sets exhibited similar composite score of arbitrary units (AU) magnitude and distribution by SERA IgG assay (99.5% specificity). (B) Specimens negative by SERA IgG exhibiting positive SERA IgM scores (99.1% specificity).

The performance of the SERA Lyme IgG and IgM panels was assessed using an independent validation set of 454 specimens positive for antibodies to B. burgdorferi by STTT (Lyme disease validation cohort) and >1,000 repertoires obtained from individuals with unknown Lyme serostatus (control validation cohort) (Table 1). The combined IgG and IgM panels yielded a positive agreement of 84.1% (95% CI, 80.1 to 87.5%; 382/454) with STTT (Fig. 3). The agreements in the discovery and validation sample sets were statistically similar (Z-test; *P* = 0.2018), indicating the panels were not overfit to the discovery group. Five of 1,076 epitope repertoires without STTT information from our database were SERA positive for IgG, yielding a specificity of at least 99.5%, and an additional 10 were SERA positive by IgM (99.1% specificity). Combining the IgG and IgM scores using a simple OR function (IgG positive or IgM positive) yielded a lower bound on specificity of 98.6% (Fig. 3). Interestingly, two of these control samples with the highest SERA IgG scores (composite scores of 390 and 123) were subsequently tested positive by STTT (10 and 6 positive bands by IgG immunoblot, respectively), suggesting that these individuals likely had prior or ongoing Lyme disease and that the SERA Lyme disease IgG assay specificity is 99.7%.

The article "Serum Epitope Repertoire Analysis Enables Early Detection of Lyme Disease with Improved Sensitivity in an Expandable Multiplex Format" was published in 2021. Journal: J Clin Microbiol.

To investigate the ability of the SERA assay to detect early Lyme disease, we compared the performance of the validated IgG and IgM panels and STTT in an additional set of clinically defined Lyme disease specimens (*n* = 119) of which a subset of these subjects are Lyme positive by culture, PCR, or additional clinical criteria, including EM (9). Among clinically defined Lyme samples, 37 were from stage 2 or 3 Lyme disease, including Lyme arthritis (*n* = 29; stage 3), neuroborreliosis (*n* = 6; stage 2), and carditis (*n* = 2; stage 2), and all were positive by both STTT and SERA. The remaining 82 samples were defined as early Lyme (stage 1), of which 45 were STTT negative and 37 were IgM STTT positive. SERA identified 22 of the 45 STTT negative samples as positive, while 4 STTT-positive samples were negative by SERA (Fig. 4A). Control cohorts, including Lyme disease lookalike samples (*n* = 78) that can cause STTT false positives, as well as non-Lyme controls (*n* = 179), were also analyzed (Table 1; Fig. 4A).

**FIG 4:** SERA provided increased sensitivity in clinically defined Lyme disease cases. The SERA IgG plus IgM Lyme assay and standard two-tier testing (STTT) were performed on clinically defined Lyme disease, including 57 matched early (acute and convalescent) samples from the Centers for Disease Control (CDC) and Lyme Disease Biobank (LDB). (A and C) STTT-negative Lyme samples from both the CDC and LDB are positive by SERA giving improved sensitivity compared to STTT while retaining equivalent specificity. (A) SERA scores for the IgG panel shown for STTT-positive and STTT-negative Lyme and non-Lyme samples from the CDC and LDB separately. (IgG-negative points in red are SERA IgM positive.) (B) Sensitivity, specificity, and accuracy of SERA and STTT IgG and IgM on combined cohorts of clinically defined Lyme samples. (*, sensitivity *P* = 0.0112, accuracy *P* = 0.0107; Z-test; error, 95% CI). (D) Sensitivities and comparison significance of SERA and STTT on matched acute and convalescent early Lyme cases.

The article "Serum Epitope Repertoire Analysis Enables Early Detection of Lyme Disease with Improved Sensitivity in an Expandable Multiplex Format" was published in 2021. Journal: J Clin Microbiol.

Compared to STTT, SERA exhibited superior sensitivity on both the CDC and Lyme Disease Biobank (LDB) cohorts, 86% versus 72% and 65% versus 48%, respectively, providing a statistically significant increase in sensitivity of 15% for all Lyme disease samples in these two cohorts (77% versus 62% for SERA versus STTT; z-test, *P* = 0.0112) (Fig. 4A to C). Significantly increased sensitivities of 26% and 19% were observed in both acute and convalescent early Lyme draws among 57 matched samples (Fig. 4D). The measured specificity of SERA in the clinically defined non-Lyme cohorts was 99%, which is not significantly different from the lower bound estimated from the validation controls (98.6%). The increased specificity of SERA relative to STTT (99% versus 97%) did not reach statistical significance.

Given the apparent improvement in sensitivity of SERA compared to STTT in two separate cohorts of clinically confirmed early Lyme disease, we more closely reviewed the specific testing status for paired acute- and convalescent-phase samples that were positive by SERA but negative by STTT. SERA IgG and IgM scores for seven acute and convalescent matched samples are provided as examples (Fig. 5). All seven specimens were positive by SERA (IgG and/or IgM) but negative by STTT at the acute draw (Fig. 5). Four of these became STTT positive on the convalescent draw, while the other three remained STTT negative (Table S3). In five of these seven matched specimens, the IgG SERA score increased at least 50% between the acute and convalescent draws, including in two of the three subjects that were negative by STTT on both draws (Table S3). These examples further support the observed improved sensitivity of SERA relative to STTT during the early stages of infection. The IgG motif panel also enabled differentiation of stages of Lyme disease. A larger number of motifs were positive for late-stage Lyme disease (Lyme arthritis) than for acute or convalescent-phase sera (Mann-Whitney U test, *P* < 0.0001). Furthermore, a subset of motifs were enriched in late Lyme disease that were absent during early stages of disease (Fig. 5).

**FIG 5:** SERA IgG motif and panel detection of clinically staged Lyme samples. (A) IgG motif enrichment of Lyme samples. Red boxed motifs indicate VlsE antigens enriched in all stages of Lyme samples. Black box shows an example motif highly enriched only in later Lyme stages. (B) Staged Lyme samples plotted by number of positive IgG motifs. (C) Example of matched acute and convalescent Lyme sample composite scores on an IgG panel (solid lines) and an IgM panel (dashed lines). Solid or open points indicate panel positive or negative respectfully for each colored sample.

The article "Serum Epitope Repertoire Analysis Enables Early Detection of Lyme Disease with Improved Sensitivity in an Expandable Multiplex Format" was published in 2021. Journal: J Clin Microbiol.

## DISCUSSION

Lyme disease diagnostic tests in clinical use suffer from poor sensitivity and specificity in the early stage of disease when antibody concentrations are low and STT serology is often dependent on IgM antibodies (7, 9). Because Lyme disease is the most common vector-borne disease in the United States (1), the low sensitivity of STTT in acute infections (as low as 29 to 40% [7, 10]) may result in up to half of the cases being missed by initial testing, with resultant disease costs in the United States estimated at $1 billion each year (24). In addition, thousands of false-positive results by the STTT algorithm lead to unnecessary antibiotic use and can delay diagnosis of other infectious and autoimmune diseases with similar symptoms (25, 26). Thus, there remains a clear need to further improve the accuracy of Lyme disease testing.

Here, we demonstrated a statistically significant improvement in sensitivity from 44% to 70% for two separate cohorts of clinically defined acute Lyme disease cases using the SERA platform. SERA identified several immunogenic epitopes in novel candidate antigens that may contribute to sensitivity. Additionally, degenerate motifs may effectively represent multiple antigenically distinct B. burgdorferi strains, thereby improving sensitivity (27) or otherwise broadening the reagent composition for detecting subtly different antibodies made by each individual. Regardless, the SERA Lyme IgG and IgM assays provide meaningful sensitivity improvements for detection of early Lyme disease.

Specificity of the Lyme disease STTT algorithm is adversely impacted by IgM antibody promiscuity on enzyme immunoassays and IgM immunoblots (11, 28). Multiple studies have reported false-positive rates of Lyme disease IgM immunoblot testing (29) as high as 30 to 50% (28, 30, 31), depending on the tested population. IgM serology is further complicated by a number of lookalike diseases (e.g., mononucleosis, syphilis, periodontitis, rheumatoid arthritis, lupus, and others), which can lead to cross-reactivity in IgM EIAs and immunoblots (9). This problem has led to the recommendation that IgM immunoblots be used only in cases of acute infection within 1 month of suspected tick bite (32). Importantly, in our validation cohort of 454 STTT-positive, presumptive Lyme samples from Mayo Clinic, 71% (51 of 72) of discordant samples were positive by STTT IgM immunoblot only, yet negative by SERA, suggestive of false-positive IgM serology. By focusing the SERA assay on well-defined epitope motifs, which may be more specific than linear peptides, we were able to achieve exceptional specificity for both the IgG (99.5%) and IgM (99.1%) assays such that they could be combined to provide excellent overall specificity (98.6%). Thus, the SERA IgG and IgM Lyme assays may significantly increase case detection while reducing false-positive rates.

The article "Serum Epitope Repertoire Analysis Enables Early Detection of Lyme Disease with Improved Sensitivity in an Expandable Multiplex Format" was published in 2021. Journal: J Clin Microbiol.

Available diagnostic tests for Lyme disease (STTT and MTTT) do not readily distinguish between the three stages, which include (i) early localized disease, (ii) early disseminated disease, and (iii) late Lyme disease (33). Yet knowledge of disease stage can be important to guide appropriate dose and duration of antibiotic therapy (34). Others have suggested that the number of positive immunoblot bands or epitopes is a useful metric to stage disease (14, 35). In accordance with this hypothesis, we observed a statistically significant increase in the number of positive motifs in cases of Lyme arthritis. While VlsE epitope-specific antibodies were evident in specimens with early disease, the number of epitopes and magnitude of response increased through stage 2 and 3 specimens. These results are consistent with reports of upregulated VlsE expression levels following infection and host immune response (36, 43).

In addition, many more stage 3 samples have strong reactivity to motifs mapping to flagellar protein components (e.g., flagellin, flagellar filament 41 kDa antigen, and flagellar M-ring protein). Interestingly, specimens from stage 3 Lyme disease exhibited reactivity toward motifs that map to B. burgdorferi proteins such as P66, MlpB, and PF-32 plasmid partition protein, which were largely absent from early Lyme samples. These observations are consistent with the hypothesis that early B. burgdorferi infection utilizes VlsE as a highly antigenic “decoy” resulting in a reduced antibody response to other surface proteins (44). A more directed discovery effort within expanded cohorts of clinically confirmed stage 2 and stage 3 patients may yield additional B. burgdorferi antigens/motif biomarkers to assess Lyme disease stage.

Although SERA has achieved a significant improvement for detection of acute early Lyme samples, 30% of these samples remain serologically negative (Fig. 4D). Our early Lyme cohorts include 13 samples that were PCR or culture confirmed (LDB cohort), of which 8 are STTT and SERA negative (the remaining 5 were STTT and SERA positive). The subjects in the CDC early Lyme cohort are designated to be at risk for *Borrelia* infection, presented with EM rash, and were confirmed by PCR and culture in most cases (8). These samples thus represent very early infection and therefore may lack sufficient antibody concentrations for detection. Only 7 STTT-negative samples were included in motif discovery; therefore, it is possible that discovery using the full set of 45 STTT-negative samples and additional samples positive only by culture (on nucleic acid testing [NAT]) could reveal additional epitope motifs that enhance the sensitivity of SERA for early Lyme infections. Even so, curated national specimen repositories have sourced modest numbers of such specimens, likely due to the paucity of cultures ordered. The panel described here could be readily updated with additional discovery efforts, should additional culture-positive (STTT-negative) specimens become available.

The article "Serum Epitope Repertoire Analysis Enables Early Detection of Lyme Disease with Improved Sensitivity in an Expandable Multiplex Format" was published in 2021. Journal: J Clin Microbiol.

Several other recently developed tests have been shown to improve sensitivity in early Lyme disease (13–15, 37, 38). For example, a point-of-care microfluidic assay (mChip-Ld) using three Lyme antigens showed a 29% and 5% improvement in sensitivity in two separate early Lyme cohorts, respectively (13). Another multiantigen test developed to improve IgM plus IgG serology demonstrated sensitivities in acute and convalescent early Lyme samples of 70% and 84%, respectively, equivalent to sensitivities of SERA (37). A recently FDA-approved bead-based Luminex assay (Bio-Rad) yielded 15% and 20% improvement in sensitivity relative to STTT in baseline and “posttreatment” early Lyme samples, respectively (38). Finally, a Serochip assay was developed to enable multiplex testing for eight tick-borne diseases (15); however, sensitivity in similarly sized cohorts of early Lyme disease was not reported. SERA, like Serochip, enables multiplex testing for any number of tick-borne diseases (and other infections) and, as shown here, provides statistically significant improvements in sensitivity in early Lyme disease, along with improved specificity.

Importantly, B. burgdorferi is just one of many pathogens transmitted by ticks (39). Considering increasing numbers of Ixodes scapularis tick vectors and their expanding geographic range, accurate diagnostic tests for tick-borne diseases are critical. Because a single SERA assay can detect an arbitrary number of antibody specificities (15), SERA is well suited for multiplex testing for any number of tick-borne pathogens in a single expandable assay. Of particular importance, *Babesia* species are often transmitted by I. scapularis with or without B. burgdorferi coinfection and require a distinct antibiotic regimen (40). Our results indicate that SERA provides a means to discover diagnostically effective epitopes, allowing development of serology tests with improved performance for many infectious diseases.

The article "Serum Epitope Repertoire Analysis Enables Early Detection of Lyme Disease with Improved Sensitivity in an Expandable Multiplex Format" was published in 2021. Journal: J Clin Microbiol.

We are developing SERA to be used without significant modification within clinical testing laboratories. We anticipate that the assay will be offered initially from a centralized Clinical Laboratory Improvement Amendments (CLIA)-certified, College of American Pathologists (CAP)-accredited laboratory. Longer-term, large commercial testing labs and state and federal labs could develop laboratory-developed tests (LDTs) within their existing CLIA labs using manufactured library reagents, published epitope and algorithm information, and available software. In the authors’ facility, the assay is routinely performed in 96-well deep-well plates and semiautomated using off-the-shelf liquid-handling instrumentation. For library quality assessment, we typically sequence 400 to 500 million library members to quantify diversity and ensure lack of bias toward particular sequences. Thus, we have not identified any barriers to routine use of SERA in the setting of a clinical testing lab.

## Supplementary Material

Supplemental file 1
